# Antimicrobial Activities and Biopreservation Potential of Lactic Acid Bacteria (LAB) from Raw Buffalo (*Bubalus bubalis*) Milk

**DOI:** 10.1155/2023/8475995

**Published:** 2023-02-07

**Authors:** Muhammad Saleem Kalhoro, Anil Kumar Anal, Dildar Hussain Kalhoro, Tarique Hussain, Ghulam Murtaza, Mazhar Hussain Mangi

**Affiliations:** ^1^Food Engineering and Bioprocess Technology, Department of Food, Agriculture & Bioresources, Asian Institute of Technology, P.O. Box 4, Pathumthani 12120, Thailand; ^2^Department of Veterinary Microbiology, Faculty of Animal Husbandry and Veterinary Sciences, Sindh Agriculture University, Tandojam 70060, Pakistan; ^3^Animal Sciences Division, Nuclear Institute for Agriculture and Biology (NIAB), P.O. Box 128, Jhang Road, Faisalabad, Pakistan; ^4^Department of Animal Reproduction, Faculty of Animal Husbandry and Veterinary Sciences, Sindh Agriculture University, Tandojam 70060, Pakistan; ^5^Key Laboratory of Animal Epidemiology and Zoonosis, Ministry of Agriculture, National Animal Transmissible Spongiform Encephalopathy Laboratory, College of Veterinary Medicine, China Agricultural University, Beijing 100193, China

## Abstract

The aim of this study was to investigate the antimicrobial and biopreservation potential of lactic acid bacteria. The potential probiotic culture inhibited the growth of gram-positive and gram-negative foodborne pathogens in agar spot assay with inhibition zones ranging from 10 to 21 mm in diameter. The strains showed coaggregation capabilities ranging from 7 to 71% with tested food pathogens including *Escherichia coli*, *Staphylococcus aureus*, *Listeria monocytogenes*, and *Salmonella enterica* subsp. *enterica* serovar Typhimurium. The effect of cell-free supernatants on the release of 260 nm absorbing material, especially nucleic acids, was evaluated and indicated the antagonistic activity on foodborne pathogens, the highest being *Lactobacillus paraplantarum* against *E. coli* (3.77) and *S. aureus* (3.86) after 60 min. The effect of cell-free supernatant (CFS) on the growth of pathogens showed that *Lactobacillus paraplantarum* 11 and *L. pentosus* 93 had the highest inhibitory activity against tested strains. The biopreservation assay indicated that the potential probiotic strains *Lactobacillus paraplantarum* 11 (BT), *Lactiplantibacillus plantarum* 19, *Lactobacillus pentosus* 42, *Limosilactobacillus fermentum* 60, *Lactobacillus pentosus* 93, and *Limosilactobacillus reuteri* 112 were effective in reducing the *Listeria monocytogenes* population in raw buffalo milk. Complete *Listeria monocytogenes* inhibition was observed after 6-8 days. This study showed that probiotic LAB from buffalo milk have antimicrobial and biopreservation potential; these strains have the potential to be utilized as biopreservative agents in food products.

## 1. Introduction

Food spoilage by microorganisms leads to significant economic losses as well as health problems [1]. Foodborne pathogens are a threat to food quality and result in several diseases and disorders such as respiratory infections, inflammatory diseases, intestinal disorders, and cancer [2]. In recent years, there has been growing interest in alternative natural ways to control food spoilage due to the harmful effects of artificial chemicals and antimicrobial resistance [3]. The prevention of food spoilage by using biopreservative agents such as probiotics and their antimicrobial compounds is a satisfactory alternative approach to prevent spoilage without altering the taste and smell of food products [4].

The lactic acid bacteria (LAB), considered potential probiotic candidates, are the diverse group of gram-positive, non-spore-forming, catalase and cytochrome oxidase negative, and nonmotile bacteria, which produce lactic acid as a product of fermentation [5, 6]. The basic criteria for the LAB strains to be used as probiotics include the following: (1) they should have GRAS status, (2) they should be resistant to low pH and high bile concentration and survive in gastrointestinal fluids, (3) they should have adhesion characteristics, (4) they should have antibacterial characteristics against enteric pathogens, and (5) they should survive and be viable during the processing and storage [7]. There are different sources of LAB such as fermented meat, fish, milk, cheese, and herbs [1, 8–11].

The LAB are associated with several health benefits such as improvement of gastrointestinal tract conditions, antibacterial and antifungal activities, antiallergic and antioxidant properties, and lowering cholesterol levels and immunomodulatory activities [12, 13]. The LAB produce their antimicrobial activity through the reduction of pathogen translocation, inhibition of pathogen adherence, and production of antimicrobial compounds [14]. Antimicrobial compounds produced by lactic acid bacteria include organic acids, hydrogen peroxide, diacetyl, and bacteriocins, which can inhibit the growth of bacteria as well as fungi [11, 14].

Increased outbreaks of foodborne diseases in recent years along with antimicrobial resistance of pathogens against commercial antibiotics [8] demand greater interest and need for natural alternative ways to control foodborne pathogens. Lactic acid bacteria and their antimicrobial metabolites can inhibit foodborne pathogens and act as natural biopreservatives. Very limited studies have been reported on biopreservative potential of the probiotics from buffalo milk and their antimicrobial metabolites [11, 13]. Therefore, the present study was undertaken to characterize the antimicrobial activity of probiotic LAB isolated from raw buffalo milk and to evaluate their biopreservation potential.

## 2. Materials and Methods

### 2.1. Indicator Pathogenic Strains

*Bacillus cereus* (ATCC 11778), *Bacillus subtilis* (*ATCC 6633*)*, Escherichia coli* (ATCC 25922), *Enterococcus faecalis* (ATCC 19433), *Listeria monocytogenes* (*ATCC 19115*), *Listeria innocua* (ATCC 33090), *Salmonella enterica* subsp. *enterica* serovar Enteritidis (ATCC 13076), *Salmonella enterica* subsp*. enterica* serovar Typhimurium (ATCC 13311), *Shigella dysenteriae (*ATCC 11835), *Staphylococcus aureus* (*ATCC 25923*), and *Pseudomonas aeruginosa* (ATCC 27853) were used as pathogenic indicator strains.

### 2.2. Probiotic Strains

*Lactobacillus paraplantarum* 11 (BT), *Lactiplantibacillus plantarum* 19, *Lactobacillus pentosus* 42, *Limosilactobacillus fermentum* 60, *Lactobacillus pentosus* 93, and *Limosilactobacillus reuteri* 112, which were previously isolated from buffalo milk were used as probiotic strains in this study [11, 13]. The strains were preserved in 20% glycerol and resuscitated in MRS broth.

### 2.3. Antibacterial Activity of Live Probiotic Culture

Antibacterial activity against foodborne pathogens was evaluated through the agar spot method as a previously described method [15] with slight modifications. The cell culture of potential probiotic strains was spotted (5 *μ*L) on MRS agar plates and incubated at 37°C for 48 h. The plates were overlaid with 10 mL of BHI soft agar (0.75% agar) which was previously inoculated with pathogens (10^4^ CFU/mL). The diameter of the inhibition zone was measured after incubation at 37°C for 24 h.

### 2.4. Coculture of Isolated Probiotics with Test Foodborne Pathogens

The coculture of probiotic strains with foodborne pathogens was determined as the previously described method [16] with slight modifications. The cell culture (500 *μ*L) of each potential probiotic and pathogenic strain was mixed (1 : 1) and incubated at 37°C for 24 h. The total plate count of indicator pathogenic strains was performed on selective agar medium (MacConkey agar for *E. coli* and Baird Parker agar for *Staphylococcus aureus*). The monoculture of pathogenic and probiotic strains was grown at 37°C for 24 h, and the total plate count was performed on selective medium, which was used as control.

### 2.5. Evaluation of Coaggregation of Isolated Probiotics with Test Pathogens

The coaggregation activity was evaluated as the previously described method [17] with slight modifications. Cell culture (500 *μ*L) of probiotic and pathogenic strains were mixed and incubated at 37°C for 24 h. The absorbance (A600nm) of the mixture and each culture probiotic and pathogenic strain alone was measured through Uv-Vis spectrophotometer (UV-1800, Shimadzu, Japan).

The coaggregation percentage was calculated by the following equation:

(1) $$\begin{array}{c} \left[\left(\text{Apat}+\text{Aprobio}\right)/2-\left(\text{Amix}\right)\right]/\left(\text{Apat}+\text{Aprobio}\right)/2\times 100\%, \end{array}$$

where Apat = absorbance (A600nm) of pathogen, Aprobio = absorbance (A600nm) of probiotic, and Amix = absorbance (A600nm) of mixture.

### 2.6. Effect of Cell-Free Supernatant on Releasing the Cellular Materials

The effect of cell-free supernatant (CFS) on the release of cellular materials from pathogens (*E. coli* and *S. aureus*) was evaluated following the previously described method [18], with slight modifications. Overnight cultures of *E. coli* and *S. aureus* were washed twice and resuspended in sterile peptone water. The overnight culture of probiotic strains was centrifuged, and CFS was collected. The CFS (1.5 mL) of probiotic strains was mixed with pathogen culture (1.5 mL) and incubated at 37°C. The cell suspensions were centrifuged (10,000 rpm for 10 min 4°C) at 0, 30, and 60 min of intervals. The supernatant was taken to measure the absorbance at OD_260_ nm using the Uv-Vis spectrophotometer (UV-1800, Shimadzu, Japan). The control was prepared the same way without the addition of CFS.

### 2.7. Effect of CFS on Growth of Pathogens

The antibacterial activity of CFS on the growth of *S*. Typhimurium, *L. monocytogenes*, *E. coli*, and *S. aureus* was evaluated by following a previously described method [19] with slight modifications. The potential probiotic strains were centrifuged (10,000 rpm for 10 min 4°C), and CFS was collected and sterilized through 0.2 *μ*m membrane filter (Sartorius, Minisart, Germany). The CFS (10 mL) of each LAB strain was mixed with 100 mL of cell culture of each pathogenic strain and incubated at 37°C for 24 h. The optical density (OD_600 nm_) was measured every 2 h through a Uv-Vis spectrophotometer (UV-1800, Shimadzu, Japan). The cell cultures of *S*. Typhimurium, *L. monocytogenes*, *E. coli*, and *S. aureus* without the addition of CFS were used as control.

### 2.8. Biopreservation Potentials of Probiotic LAB in Raw Milk

The biopreservation potential of probiotic LAB strains against *L*. *monocytogenes* in buffalo milk was performed following the previously described method [20] with slight modifications. Pasteurized buffalo milk (50 mL) samples were inoculated with 1 mL of *L*. *monocytogenes* and probiotic culture. The milk samples were stored for 10 days at 37°C. The samples were drawn every day, and the total plate count was performed on Listeria selective agar and MRS agar (HiMedia, India). The samples containing *L*. *monocytogenes* culture were used as control.

### 2.9. Statistical Analysis

Data are presented as the mean and standard deviation (mean ± SD) of three independent replicates. Statistical analysis was performed using the SPSS 23.0 program (SPSS Inc., Chicago, IL).

## 3. Results and Discussion

Very limited studies have been reported on probiotics and their antimicrobial effects from buffalo milk and their antimicrobial effects on pathogens. In this study, the effect of live culture of probiotics and their CFS on the growth of pathogenic bacteria is observed. The probiotic culture was used as a biopreservative in order to improve the shelf life of fermented milk products. Purification and characterization of antimicrobial compounds were not performed as the major objective of this research was to use live LAB culture as an inhibitory substance. One isolate (*L*. *paraplantarum* BT-11) produced bacteriocin-like inhibitory substance (BLIS), which has been already reported by the main author [13]. Live culture of LAB and their CFS were used against both gram-positive and gram-negative pathogens in several experiments during this study including the biopreservation test to further explore the inhibitory potential of probiotic LAB.

### 3.1. Antibacterial Activity of Live Cells

The antibacterial activity of live cells of LAB against foodborne pathogens is shown in Table 1. All probiotic strains displayed antagonistic activity against tested indicator pathogens in the agar spot assay. The live culture probiotic strains showed antagonistic activity against both gram-positive (*B cereus*, *B. subtilis*, *L. monocytogenes*, *L. innocua*, and *S. aureus*) and gram-negative (*E. coli*, *Enterococcus faecalis*, *S. Enteritidis*, *S.* Typhimurium, *Shigella dysenteriae*, and *P. aeruginosa*) pathogens. The inhibitory activity ranged from 10 to 21 mm. *L. paraplantarum* 11 (BLIS-producing strain) produced the highest antibacterial activity against *L. monocytogenes*.

The antagonistic activity of LAB or their antimicrobial compounds is an important characteristic of probiotics. The probiotic bacteria produce several compounds such as organic acids (lactic acid, acetic acid, and butyric acid), hydrogen peroxide, and bacteriocins or BLIS which shows the antagonistic activity against the pathogens [21]. Palachum et al. [10] reported antibacterial activity of live culture of probiotic strain *L. plantarum* WU-P19 against gram-positive and gram-negative pathogens. The antibacterial activity of the live cultures in the present study was higher than that reported by Monteagudo-Mera et al. [22].

### 3.2. Coculture with Pathogens

Table 2 represents the coculture of pathogens with probiotics. The survival of *E. coli* and *S. aureus* was 4.1 to less than 3 Log CFU/mL and 3.9 to less than 3 Log CFU/mL and 5 to 6 Log CFU/mL reduction in coculture with probiotic strains. Coculture studies of probiotics and pathogens help to understand the effects of probiotics on the growth of foodborne pathogens. Afolayan and Ayeni [16] reported 6 Log CFU/mL reduction of *E. coli* after coculture with *L. plantarum* and *L. fermentum*. In a similar study, Voravuthikunchai et al. [23] reported inhibitory activity of *L. reuteri* (L22) against MRSA with 4 Log CFU/mL survival and complete inhibition of *S. aureus* after 24 h incubation in coculture experiment. Drago et al. [24] reported 4-5 and 6 Log CFU/mL reduction in the population of *E. coli* and *S*. Enteritidis, respectively, after coculture study with Lactobacilli strains. The difference in MRS medium, which contains complex proteins, may also affect the growth of strains in coculture studies [25].

### 3.3. Coaggregation with Pathogens

The coaggregation activity of probiotic LAB with *E. coli*, *S*. Typhimurium, *S*. *aureus*, and *L. monocytogenes* is shown in Figure 1. All probiotic isolates exhibited coaggregation with pathogens. *L. paraplantarum* (BT-11) showed the highest coaggregation percentage (71%) against *S. aureus* whereas the lowest coaggregation percentage (7%) was shown by *L. reuteri* (112) against *E. coli*. The coaggregation capability of probiotics with pathogens is a good indicator of their gut colonization property. Coaggregation with pathogens enhances the probiotic potential and cellular aggregation that promote the colonization of probiotic bacteria [26, 27]. Kumari et al. [28] reported the coaggregation ability of LAB strains isolated from fermented foods and beverages with *L. monocytogenes* (11-72%).

### 3.4. Effect of CFS on 260 nm Releasing Materials

The effect of CFS of LAB strains on the release of *E. coli* and *S. aureus* 260 nm absorbing material (DNA and RNA) is shown in Tables 3 and 4. The absorbance values increasing at an optical density of 260 nm with time indicate the cell death of indicator pathogenic strains while control for both strains remained the same. The release of the extracellular material indicates the integrity of the cell membrane; nucleotides (DNA, RNA) absorb ultraviolet light at 260 nm; therefore, they are termed 260 nm absorbing materials [29]. The release of 260 nm absorbing material (DNA and RNA) due to the CFS of probiotic strains leads to the loss of essential cell electrolytes and cell structure and integrity [8]. Different antimicrobial compounds are reported to produce their antagonistic activity through leakage of cytoplasm and its coagulation, which affects the functions and integrity of the affected cell leading to cell death [30]. Similar results regarding the loss of 260 nm absorbing materials of pathogens due to the antimicrobial compounds or LAB were also reported [8, 31, 32].

### 3.5. Effect of CFS on Growth of Foodborne Pathogens

Figures 2–5 illustrate the antibacterial activity of *L*. *paraplantarum* 11, *L. plantarum* 19, *L. pentosus* 42, *L. fermentum* 60, *L. pentosus* 93, and *L. reuteri* 112 on the growth of foodborne pathogens. The results show the reduction in the growth of pathogenic strains with the addition of CFS. All probiotic strains had a broad antimicrobial spectrum against the growth of gram-positive and gram-negative pathogens. The CFS of isolate *L*. *paraplantarum* 11 and *L. pentosus* 93 revealed the highest antibacterial activity against all indicator strains. The antimicrobial activity of CFS can be attributed to the presence of several antimicrobial compounds such as organic acids, hydrogen peroxide, reuterin, reutericyclin, bacteriocin, or BLIS. These results indicate the antimicrobial characteristics of potential probiotic strains and their potential to be used in several food and biomedical applications. Ahmadova et al. [33] reported bacteriostatic antibacterial effect of LAB strain *E. faecium* AQ71 from cheese against *L. monocytogenes* and bactericidal effect against *Levilactobacillus brevis* while Khodaei and Sh [19] reported reduced growth of *P. aeruginosa* and *L. monocytogenes* after the addition of CFS of enterococci in a similar experiment.

### 3.6. Biopreservation in Milk

Figure 6 illustrates the antibacterial effects of six probiotic strains in raw buffalo milk against *L. monocytogenes*. The results show that the probiotic strains have a biopreservative effect on raw milk against *L. monocytogenes*. The growth of *L. monocytogenes* was gradually reduced with time as compared to the control. The probiotic LAB strains showed an antagonistic effect against *L. monocytogenes* in raw buffalo milk. No growth of *L. monocytogenes* was found after the 6^th^ day (*L. paraplantarum* 11, *L. pentosus 42*, and *L. pentosus* 93), 7^th^ day (*L. plantarum* 19, *L. reuteri* 112), and 8^th^ day (*L. fermentum* 60).

In this study, the effect of live culture of potential probiotic LAB was performed as a challenge study. Live cultures of probiotic LAB were used to compare the effects of longer storage periods on the growth of LAB and pathogenic bacteria (in terms of Log CFU/mL) in milk. Fermented milk showed a reduction in the growth of pathogenic bacteria during the storage period. Lactic acid bacteria and their antimicrobial compounds are used as biopreservatives. One of the objectives of this study was to compare the increase in the growth of LAB and decrease in the growth of pathogens in fermented milk with longer storage periods; with CFS or purified compounds, this comparison was not possible; therefore, live cultures of LAB were used for the biopreservation purpose. Fernandes et al. [20] also reported a similar study of control of *L. monocytogenes* in raw milk through *L. plantarum* culture.

The LAB are most suitable candidates for biopreservation as they are naturally present in many food products and produce antimicrobial compounds against pathogens [34]. The probiotic strains isolated from the same source where they will be used as biopreservative agents are more preferred as they have adopted the rough environmental conditions of that food product and are more competitive than LAB strains from other sources [35].

Several studies have reported the biopreservation potential of LAB in foods against foodborne pathogens [36, 37]. *L. monocytogenes* growth was inhibited in whole milk with antimicrobial compounds produced by *Lactobacillus curvatus* [38]. Sriwattanachai et al. [39] reported food preservation potential and synergistic effect of *L. plantarum* CFS and essential oil. Akbar and Anal [40] reported complete inhibition of *S. aureus* in poultry meat with *L. lactis* culture.

## 4. Conclusion

A detailed study was conducted on the antimicrobial and biopreservation potential of probiotics from buffalo milk. Six probiotic LAB strains (*L. paraplantarum* 11, *L. plantarum* 19, *L. pentosus* 42, *L. fermentum* 60, *L. pentosus* 93, and *L. reuteri* 112) showed promising antibacterial and biopreservation potential. Live cultures of all strains were effective in reducing the growth of foodborne and spoilage-causing pathogens. The viable count of gram-positive and gram-negative pathogens was reduced in the coculture assay. The probiotic strains showed aggregation characteristics; the CFS had a significant effect on pathogens, which was reflected by the release of 260 nm absorbing material and reduced growth of pathogens. The live culture of probiotic strains showed biopreservative potential against *L. monocytogenes* in raw milk. Based on the results, the potential probiotic strains have the potential to be used as natural biopreservative agents against foodborne pathogens.

## Figures and Tables

**Figure 1:** Coaggregation activity of *L. paraplantarum* 11, *L. plantarum* 19, *L. pentosus* 42, *L. fermentum* 60, *L. pentosus* 93, and *L. reuteri* 112 strains with pathogenic strains after incubation at 37°C for 24 h. Mean ± SD of three independent readings.

**Figure 2:** Effect of cell-free supernatant (CFS) of *L. paraplantarum* 11, *L. plantarum* 19, *L. pentosus* 42, *L. fermentum* 60, *L. pentosus* 93, and *L. reuteri* 112 on the growth of *S.* Typhimurium during 24 h incubation at 37°C. The *S.* Typhimurium culture without CFS was used as control. Mean ± SD of results from three replicates.

**Figure 3:** Effect of cell-free supernatant (CFS) of *L. paraplantarum* 11, *L. plantarum* 19, *L. pentosus* 42, *L. fermentum* 60, *L. pentosus* 93, and *L. reuteri* 112 on the growth of *L. monocytogenes* during 24 h incubation at 37°C. The *L. monocytogenes* culture without CFS was used as control. Mean ± SD of results from three replicates.

**Figure 4:** Effect of cell-free supernatant (CFS) of *L. paraplantarum* 11, *L. plantarum* 19, *L. pentosus* 42, *L. fermentum* 60, *L. pentosus* 93, and *L. reuteri* 112 on the growth of *E. coli* during 24 h incubation at 37°C. The *E. coli* culture without CFS was used as control. Mean ± SD of results from three replicates.

**Figure 5:** Effect of cell-free supernatant (CFS) of *L. paraplantarum* 11, *L. plantarum* 19, *L. pentosus* 42, *L. fermentum* 60, *L. pentosus* 93, and *L. reuteri* 112 on the growth of *S. aureus* during 24 h incubation at 37°C. The *S. aureus* culture without CFS was used as control. Mean ± SD of results from three replicates.

**Figure 6:** Biopreservation effect (0) of *L. paraplantarum* 11 (a), *L. plantarum* 19 (b), *L. pentosus 42* (c), *L. fermentum* 60 (d), *L. pentosus* 93 (e), and *L. reuteri* 112 (f) against *L. monocytogenes* in milk during 10 days of storage. The samples containing *L. monocytogenes* culture were used as control (black diamond). Mean ± SD of three independent readings.

**Table 1:** Antibacterial activity of LAB against pathogens.

Pathogenic bacteria	Probiotic strains					
	11	19	42	60	93	112
	Diameter of inhibition zone (mm)					
*B. cereus*	16.3 ± 0.5	15.0 ± 0.0	18.3 ± 0.5	15.3 ± 0.5	17.6 ± 0.5	14.0 ± 0.0
*B. subtilis*	15.3 ± 0.5	17.3 ± 0.5	16.3 ± 0.5	13.0 ± 0.0	14.3 ± 0.5	16.3 ± 0.5
*E. coli*	19.0 ± 0.0	17.0 ± 0.0	17.0 ± 0.0	16.6 ± 0.5	19.3 ± 0.5	18.3 ± 0.5
*E. faecalis*	17.0 ± 1.0	16.0 ± 1.0	19.3 ± 0.5	18.0 ± 0.0	17.0 ± 0.0	19.6 ± 0.5
*L. monocytogenes*	21.3 ± 0.5	19.0 ± 0.0	20.3 ± 0.5	18.3 ± 0.5	18.6 ± 0.5	17.3 ± 0.5
*L. innocua*	19.6 ± 0.5	19.3 ± 0.5	17.3 ± 0.5	17.6 ± 0.5	18.6 ± 0.5	19.3 ± 0.5
*S.* Enteritidis	20.3 ± 0.5	18.0 ± 1.0	18.3 ± 0.5	19.0 ± 1.0	20.6 ± 0.5	16.6 ± 0.5
*S.* Typhimurium	20.0 ± 0.0	17.0 ± 0.0	16.6 ± 0.0	18.0 ± 0.0	19.6 ± 0.5	18.3 ± 0.5
*S. dysenteriae*	16.6 ± 0.5	17.6 ± 0.5	16.6 ± 0.5	16.0 ± 1.0	17.3 ± 0.5	17.0 ± 1.0
*S. aureus*	17.3 ± 0.5	18.0 ± 0.0	20.3 ± 0.5	19.6 ± 0.5	20.0 ± 0.0	19.0 ± 1.0
*P. aeruginosa*	16.6 ± 0.5	15.3 ± 0.5	14.3 ± 0.5	10.0 ± 0.0	16.3 ± 0.5	15.3 ± 0.5

Mean ± SD of results from three replicates. *L. paraplantarum* (11), *L. plantarum* (19), *L. pentosus* (42), *L. fermentum* (60), *L. pentosus* (93), and *L. reuteri* (112).

**Table 2:** Coculture of probiotic strains with *E. coli* and *Staphylococcus aureus* (growth in Log CFU/mL).

Isolate	LAB	*E. coli*
11	9.13 ± 0.05 (9.18 ± 0.06)	3^∗^ (9.39 ± 0.03)
19	9.11 ± 0.04 (9.30 ± 0.03)	3.82 ± 0.09 (9.40 ± 0.03)
42	9.33 ± 0.03 (9.41 ± 0.03)	4.01 ± 0.06 (9.35 ± 0.03)
60	9.02 ± 0.05 (9.21 ± 0.03)	3.74 ± 0.06 (9.41 ± 0.03)
93	9.34 ± 0.03 (9.41 ± 0.03)	3.71 ± 0.07 (9.40 ± 0.03)
112	9.05 ± 0.03 (9.10 ± 0.04)	4.17 ± 0.03 (9.40 ± 0.03)
Isolate	LAB	*S. aureus*
11	9.10 ± 0.05 (9.15 ± 0.05)	3^∗^ (9.30 ± 0.04)
19	9.19 ± 0.04 (9.22 ± 0.04)	3^∗^ (9.40 ± 0.03)
42	9.21 ± 0.04 (9.38 ± 0.03)	3.93 ± 0.05 (9.41 ± 0.03)
60	9.11 ± 0.04 (9.18 ± 0.03)	3.74 ± 0.06 (9.34 ± 0.03)
93	9.28 ± 0.03 (9.38 ± 0.03)	3^∗^ (9.34 ± 0.03)
112	9.08 ± 0.04 (9.18 ± 0.04)	3.93 ± 0.04 (9.41 ± 0.03)

Values in parentheses represent growth of controls. An asterisk (∗) indicates less than 3 value. Mean ± SD of results from three replicates. *L. paraplantarum* 11, *L. plantarum* 19, *L. pentosus* 42, *L. fermentum* 60, *L. pentosus* 93, and *L. reuteri* 112.

**Table 3:** Effect of CFS on 260 nm releasing material (nucleic acid) of *E. coli* at different time intervals.

Isolate	Time (min)	Control (OD_260 nm_)	Treatment (OD_260 nm_)
11	0	1.36	1.38
	30	1.36	2.90
	60	1.37	3.77

19	0	1.32	1.33
	30	1.34	2.25
	60	1.35	3.72

42	0	1.35	1.37
	30	1.36	2.66
	60	1.38	3.51

60	0	1.34	1.33
	30	1.37	2.85
	60	1.38	3.63

93	0	1.36	1.38
	30	1.37	2.39
	60	1.37	3.38

112	0	1.36	1.44
	30	1.38	2.48
	60	1.39	3.62

CFS = cell-free supernatant; control = *E. coli* culture; treatment = *E. coli* culture with LAB CFS. *L. paraplantarum* 11, *L. plantarum* 19, *L. pentosus* 42, *L. fermentum* 60, *L. pentosus* 93, and *L. reuteri* 112.

**Table 4:** Effect of CFS on 260 nm releasing material (nucleic acid) of *S. aureus* at different time intervals.

Isolate	Time (min)	Control (OD_260 nm_)	Treatment (OD_260 nm_)
11	0	1.42	1.46
	30	1.44	2.90
	60	1.46	3.86

19	0	1.45	1.47
	30	1.45	2.60
	60	1.47	3.43

42	0	1.44	1.48
	30	1.44	2.50
	60	1.47	3.74

60	0	1.45	1.46
	30	1.45	2.13
	60	1.46	3.60

93	0	1.42	1.44
	30	1.44	2.71
	60	1.45	3.69

112	0	1.43	1.49
	30	1.45	2.95
	60	1.46	3.72

CFS = cell-free supernatant; control = *S. aureus* culture; treatment = *S. aureus* culture with LAB CFS. *L. paraplantarum* (11), *L. plantarum* (19), *L. pentosus* (42), *L. fermentum* (60), *L. pentosus* (93), and *L. reuteri* (112).

## Data Availability

The data used to support the findings of this study are included within the article.
